This article has been retracted.

# IFN-*γ* induces PD-L1 through p38/JNK/ERK signaling pathways and counteracts the tumor promoting effect mediated by PD-L1 in Glioblastoma

**DOI:** 10.1155/2022/5492602

**Published:** 2022-06-29

**Authors:** Huafang Jia, Xiaoli Xie, Long Wang, Lijuan Wang, Fengyuan Che

**Affiliations:** ^1^Department of Neurology, Linyi People's Hospital, Qingdao University, Qingdao 266071, Shandong, China; ^2^Central Laboratory, Linyi People's Hospital, Linyi 276000, Shandong, China

## Abstract

Glioblastoma is the most malignant primary glioma. Conventional treatment methods that include surgery, radiotherapy, and chemotherapy have a limited curative effect on the tumor. With the deepening of molecular biology research, molecular targeted therapy has opened a new era of tumor therapy. Programmed death ligand 1 (PD-L1) has been proved to play a pivotal role in the tumor immune evasion process. Previous studies have confirmed the specific expression of PD-L1 in glioblastoma tissues and cells, but there are few studies on inflammation regulating PD-L1 in glioblastoma. In this study, real-time PCR, flow cytometry, and western blot were applied to detect PD-L1 in glioblastoma cells. Short hairpin RNA was used to knock down PD-L1 in glioblastoma cells. Cell counting kit-8 experiment and wound-healing assay were used to detect the proliferation and migration of glioblastoma cells. Here we demonstrated that PD-L1 was overexpressed in glioblastoma cells, and interferon-gamma (IFN-*γ*) induces PD-L1 in glioblastoma cells via activating p38/JNK/ERK signaling pathways. To summarize, PD-L1 promotes the occurrence and development of glioblastoma. IFN-*γ* counteracts the tumor-promoting effects mediated by PD-L1 in glioblastoma. IFN-*γ* regulates PD-L1 through multiple signaling pathways, but the total effect of IFN-*γ-*mediated inflammatory signals still need to be further explored in glioblastoma. PD-L1 enhances the proliferation and migration of glioblastoma cells by regulating CDK4, CDK6, MMP-2, and vimentin molecules. Most importantly, targeting PD-L1 can be applied in the treatment of glioblastoma. We speculate that IFN-*γ* may affect glioblastoma through other pathways, and we will continue to further explore the mechanisms in the future.

## 1. Introduction

Glioblastoma is one of the malignant brain tumors with the highest incidence, accounting for almost 25% of primary central nervous system tumors and 50% of adult glioma [1, 2]. At present, surgical resection and chemoradiotherapy are still the main treatment methods for glioblastoma, but the postoperative recurrence rate remains high because of its high invasiveness and invasive growth of tumor tissue [3]. Hundreds of clinical trials have been carried out for decades in glioblastoma. Nevertheless, the results of some large phase III international clinical trials show that various treatment methods have no significant effect on glioblastoma patients, and the curative effects of multiple preventive and therapeutic drugs are not ideal or have great toxic and side effects [4]. Therefore, the treatment of malignant glioma especially glioblastoma confronts great challenges. It is urgent to delve into new treatment schemes to curb the progress of glioblastoma, and further improve the prognosis of glioblastoma patients.

With the deepening of the research on tumor immune evasion, researchers gradually realize that the immune plays a significant part in preventing tumors and promoting the escape of tumor cells. Programmed death ligand 1 (PD-L1) produces inhibitory signals by binding with receptor molecules on T lymphocytes a member of immunosuppressive costimulatory molecules, which is essential for maintaining host self-tolerance and regulating innate and adaptive immunity. Interferon-gamma (IFN-*γ*) is a cytokine with multiple activities, which has been recognized as significant pleiotropy in many inflammatory processes. In previous malignant tumor studies, the tumor microenvironment can advance tumor immune escape by releasing IFN-*γ* to stimulate PD-L1 in tumor cells [5, 6]. PD-1/PD-L1 inhibitors are widely available for tumor immunotherapy, but their mechanism in glioblastoma remains uncertain.

In this article, we confirmed that PD-L1 was expressed in glioblastoma cells. IFN-*γ* upregulated the expression of PD-L1 by activating p38/JNK/ERK signaling pathways. PD-L1 knockdown suppressed the proliferation and migration of glioblastoma cells.

## 2. Materials and Methods

### 2.1. Cell Culture and IFN-*γ* Stimulation

Glioblastoma cell lines U251, TG-905, and A172 were cultured in the Dulbecco's modified eagle medium (DMEM; Hyclone, USA) containing 10% fetal bovine serum (FBS; Gibco, USA) and 1% penicillin/streptomycin (Gibco, USA) at 37°C, 5% CO_2_ conditions in the incubator. Fresh glioblastoma multiforme tissue, obtained from neurosurgical patients who seek medical advice in Linyi People's Hospital, was washed and cut, digested with Trypsin (USA), and filtered out tissue fragments. Pelleted cells were cultured after centrifugation to obtain primary cells (PT-1 and PT-2). All the patients signed a written informed consent form. With DMSO as control, SB203580, SP600125, and U0126 (Calbiochem, La Jolla, CA) were added to the medium. IFN-*γ* (R＆D Systems, USA) was diluted to 50 ng/mL with DMEM medium for cell stimulation after 30 min. Cells were detected at different time points.

### 2.2. Short Hairpin RNA (shRNA) and Transfection

Lentiviral-shRNA-PD-L1 and Lentiviral-shRNA-control were purchased from Santa Cruz Biotechnology (USA). Glioblastoma cells were categorized as wild type (wt) group, control-shRNA-transfected (shRNA-ctl) group, and PD-L1-shRNA-transfected (shRNA-PD-L1) group. U251, TG-905, A172, and PT-2 were cultured in six-well plates and transfected with shRNA-ctl and shRNA-PD-L1 after cell count reached 50% fusion rate according to the manufacturer's protocol. Then we used puromycin (5 *μ*g/mL) thrice to screen the cells.

### 2.3. RNA Extraction, cDNA Preparation, and Quantitative Real-Time Polymerase Chain Reaction (qRT-PCR)

The RNA of glioblastoma cells was extracted with Trizol reagent (Invitrogen, USA). RNA was reverse transcribed into cDNA using the All-in-One First-Strand cDNA Synthesis Kit (GeneCopoeia, USA) according to the manufacturer's protocol. Use the All-in-One qRT-PCR Mix (GeneCopoeia, USA) for qRT-PCR detection. The mRNA levels of PD-L1 were calculated by the 2^−△△CT^ method normalized to the Actin beta (ACTB) levels. The primers used in this research were PD-L1, 5′-GCTATGGTGGTGCCGACTAC-3′ (forward) and 5′-CACTGCTTGTCCAGATGACTTC-3′ (reverse); ACTB, 5′-TCATTCCAAATATGAGATGCGTTGT-3′ (forward) and 5′-GCTATCACCTCCCCTGTGTG-3′ (reverse).

### 2.4. Flow Cytometry Analysis

We used direct immunofluorescence of antibodies against PD-L1 to detect the expression of PD-L1 molecules on the cell surface. After being stained with antibodies for 30 min under the protection from the light condition, cells were resuspended in phosphate-buffered saline. Flow cytometry was performed using a FACS Canto. The data were analyzed by FlowJo software.

### 2.5. Cell Counting Kit-8 (CCK-8) Assay

Glioblastoma cells were cultured for 24, 48, and 72 h. The read absorbance value at 450 nm after CCK-8 (Bestbio, Shanghai, China) was put to cells.

### 2.6. Western Blot Analysis

We used a protein extraction kit (BestBio, Shanghai, China) to extract total protein and the total protein content was measured by the BCA method. Protein was isolated and prepared using 10% SDS-PAGE and PVDF membranes. The prepared membrane was blocked with 5% evaporated milk and a primary antibody (1:1000) was added and incubated overnight at 4°C. A secondary antibody (1:2000) was added and incubated with the membrane for 1 h after three washes with TBST buffer. Finally, membranes were exposed to a chemiluminescence imaging system after developing with ECL luminescent reagent. Antibodies against PD-L1 (e Bioscience, USA), GAPDH (Proteintech, USA), CDK4, CDK6, MMP-2 (Cell Signaling Technology, USA), and vimentin (Abcam, UK) were added.

### 2.7. Wound-Healing Assay

Glioblastoma cells were implanted in six-well plates until they reached 100% confluence. Then, the cell layers were scratched with the tip of the pipette (200 *μ*L) and washed with PBS to remove the cell fragment. About 2 mL of serum-free DMEM medium was added to the six-well plates and incubated at 37°C in 5% CO_2_. Samples were taken at different time points, and three scratches were randomly selected under the microscope to take photos. The results were measured by Image J software.

### 2.8. Statistical Analysis

All experimental data were performed using Graphpad Prism 8.0 software statistically. Data in every group were expressed with mean ± standard deviation (mean ± SD) and verified by three independent experiments. The difference was analyzed using *t*-test. *P* < 0.05 were defined as statistically significant.

## 3. Results

### 3.1. PD-L1 Was Expressed in Glioblastoma Cell and IFN-*γ* Enhances PD-L1 mRNA, Surface Protein, and Total Protein Expression in Glioblastoma Cells

To evaluate the expression of PD-L1 in human glioblastoma cells, we applied western blotting and flow cytometry to assess human glioblastoma cell lines (U251, TG-905, and A172) and primary tumor cells separated from tissues of glioblastoma patients (PT-1 and PT-2). The results showed that the total protein (Figure 1(a)) and surface protein levels (Figure 1(b)) of PD-L1 were expressed in the glioblastoma cells. Furthermore, we further explored the regulatory mechanisms of IFN-*γ*- (50 ng/mL) induced PD-L1 expression in glioblastoma. IFN-*γ* induced the total protein levels (Figure 1(c)) of PD-L1 in U251, TG-905, and PT-2, and the effect is the most significant at 24 h. IFN-*γ* upregulated the surface protein levels (Figure 1(c)) expression of PD-L1 in U251, TG-905, A172, PT-1, and PT-2.

### 3.2. IFN-*γ* Regulates PD-L1 Expression via the p38/JNK/ERK Signaling Pathways

Next, we elucidated the mechanism of IFN-*γ* regulating PD-L1. After treatment with SB203580, SP600125, and U0126, we performed western blotting to investigate alterations in PD-L1, p38, JNK, and ERK. The results show that blocking p38 (Figure 2(a)), JNK (Figure 2(b)), and ERK (Figure 2(c)) signaling pathways can inhibit the upregulation of PD-L1 by IFN-*γ*.

### 3.3. PD-L1 Knockdown in Glioblastoma Cells

We knocked down PD-L1 expression in glioblastoma cells via transfection of shRNA-PD-L1. The knockdown efficiency at the mRNA level was significant when comparing the shRNA-PD-L1 group with the shRNA-ctl group and wt group ( ^*∗*^ ^*∗*^ ^*∗*^*P* < 0.001,  ^*∗*^ ^*∗*^ ^*∗*^*P* < 0.001,  ^*∗*^ ^*∗*^*P* < 0.01; Figure 3(a)). Compared with the shRNA-ctl group and wt group, the expression of PD-L1 protein in the shRNA-PD-L1 group decreased (Figure 3(b)). After being stimulated with IFN-*γ*, the expression level of PD-L1 mRNA increased in the three groups ( ^*∗*^ ^*∗*^ ^*∗*^*P* < 0.001,  ^*∗*^ ^*∗*^ ^*∗*^*P* < 0.001,  ^*∗*^ ^*∗*^ ^*∗*^*P* < 0.001) by qRT-PCR (Figure 3(a)). Western blot confirmed that the expression of PD-L1 was elevated in three groups, but the expression level of PD-L1 in the shRNA-PD-L1 group was weaker than that in the shRNA-ctl and wt groups (Figure 3(b)).

### 3.4. PD-L1 Knockdown Inhibits Glioblastoma Cells Proliferation and Migration

We explored the effects of PD-L1 knockdown on glioblastoma cell proliferation and migration. These results of CCK8 assay showed that compared with the shRNA-ctl group, shRNA-PD-L1 inhibited the proliferation of U251 cells and PT-2 cells (Figures 4(a) and 4(b),  ^*∗*^ ^*∗*^ ^*∗*^*P* < 0.001). After 24 h of IFN-*γ* stimulation, the results show that there was no discernible difference in the proliferation of U251 cells (Figure 4(a)) and TG-905 cells (Figure 4(b)). A wound-healing assay was performed to examine PD-L1 in glioblastoma cell migration. The results show that there was no difference in the three groups' cell motility of U251 and TG-905 groups after 24 h. Compared with the shRNA-ctl group, the motility of U251 and TG-905 cells (Figure 5, ^*∗*^*P* < 0.05) in the shRNA-PD-L1 group decreased. After 24 and 48 h of IFN-*γ* stimulation, the results show that there was no obvious change in the migration of U251 and TG-905 cells (Figure 5).

### 3.5. PD-L1 Regulates CDK4, CDK6, MMP-2, and Vimentin Expression

To explore the specific mechanism of PD-L1 regulating glioblastoma cell proliferation and migration, we detected the expression of related protein molecules in U251 cells by using western blot. The results show that PD-L1 knocked down suppressed the expression of CDK4, CDK6, MMP-2, and vimentin. Compared with no IFN-*γ* stimulation, the expression levels of CDK4, CDK6, MMP-2, and vimentin in wt, shRNA-ctl, and shRNA-PD-L1 cells decreased after the addition of IFN-*γ* 48 h (Figure 6).

## 4. Discussion

Glioblastoma is the most invasive brain tumor, also known as glioblastoma multiforme. The high invasiveness of glioblastoma cells leads to tumor reappearance and poor prognosis [7]. At present, it is considered that surgery combined with chemotherapy or immunotherapy promotes overcoming drug resistance and improves the survival rate of glioblastoma patients [8]. Although temozolomide (TMZ), lomustine, carmustine, and bevacizumab already have Food and Drug Administration (FDA) approval to treat glioblastoma, their efficacy is very limited [9]. Most clinical trials show that drug resistance to glioma treatment remains a major obstacle, albeit great progress has been made in various cancer treatments [10]. In recent years, tumor molecular targeted therapy has become a research hotspot. However, the tumor immune molecular mechanisms driving glioblastoma remain largely elusive. Therefore, it is significant to deeply explore the specific mechanism of the occurrence and development of glioblastoma, which is of great significance for the molecular targeted therapy of glioblastoma. PD-1/PD-L1 axis plays a crucial role in tumor immunity escapes, making it an effective target of antitumor immunity. PD-L1 inhibitors have been widely used in several tumor immunotherapy, but their mechanisms in glioma remain unclear. It is known that PD-L1 in many tumors has high expression, including lung cancer, colorectal cancer, gastric cancer, melanoma, leukemia, stromal tumor, multiple myeloma, esophageal, ovarian, pancreatic, renal cell carcinoma, oral squamous cell carcinoma, and nasopharyngeal carcinoma [11–18].

Previous researchers have detected abnormal expression of PD-L1 in human glioma specimens [19], and the expression level of PD-L1 in human glioma tissues was significantly higher than that in normal brain tissue around or far away from the tumor [20]. According to a study, the expression of PD-L1 was related to the grade and genotype of glioma [21]. Compared with isocitrate dehydrogenase wild type glioma, the expression of PD-L1 was lower in isocitrate dehydrogenase mutant glioma [22]. Now a study suggests that higher serum soluble PD-L1 and soluble PD-1 are present in patients with advanced tumors, which may be potential biomarkers for prognosis in glioma patients [23]. The changes of sPD-L1 can be measured in patients using bevacizumab, and there are difference between WHO grade II-III glioma and glioblastoma [24]. The results of some research scholars show that HIF-1*α* inhibitor and anti-PD-L1 antibody combination therapy have a further effect on tumor-fighting than a single treatment in the glioma mouse model [25]. The combination of p38 MAPK inhibitor and PD-L1 antibody can prolong the survival time of GBM mice with resistant TMZ [26]. A recent study shows that orphan nuclear receptor TLX leads to immunosuppression via transcriptional activation of PD-L1 binding to PD-1 on tumor-infiltrating lymphocytes and tumor-associated macrophages in glioma [27].

We detected the expression of PD-L1 in three glioblastoma cells. The results reveal that PD-L1 was overexpressed in U251, TG-905, A172, PT-1, and PT-2 cells, which was basically consistent with previous studies. To further seek the role and mechanism of PD-L1 in the occurrence and development of glioblastoma, we found that knocking down PD-L1 in glioblastoma cells inhibited CDK4, CDK6, MMP-2, and vimentin molecular proteins, and decreased the proliferation and migration ability of glioblastoma cells. The result identifies with previous research outcomes [28], which suggests that PD-L1 may contribute to the proliferation and migration of glioblastoma cells by regulating the expression of CDK4, CDK6, MMP-2, and vimentin.

As a proinflammatory cytokine with multiple activities, IFN-*γ* plays a significant part in innate and adaptive immune responses [29]. IFN-*γ* has been confirmed to induce tumor cell apoptosis, tumor dormancy, and immune editing [30]. Initially, the researchers found that IFN-*γ* can enhance the killing effect of immune cells on the tumor by promoting Th1 cells differentiation and CTL cells activation, and prevent tumor cell proliferation and apoptosis by binding with IFN-*γ* receptors. However, there is increasing evidence that IFN-*γ* plays a related immunomodulatory role in two aspects [31]. IFN-*γ* is the strongest cytokine regulating PD-L1. Therefore, exploring the mechanism of IFN-*γ* regulating PD-L1 in tumorigenesis and development has potential clinical value. Earlier work has explored that IFN-*γ* promotes the expression of PD-L1 in tumor cells through multiple signal pathways, including PI3K/AKT, JAK/STAT, and ERK/JAK [32–34].

We detected the signal pathway-related molecular proteins downstream of IFN-*γ*. The results showed that IFN-*γ* induces hyperphosphorylation of p38, JNK, and ERK. After inhibiting the activation of the signaling pathway with SB203580, SP600125, and U0126, PD-L1 protein expression in glioblastoma cells decreased significantly. The above results show that IFN-*γ* upregulates PD-L1 expression via p38/JNK/ERK signaling pathways. IFN-*γ* with p38/JNK/ERK signaling pathways may regulate PD-L1 and promote the molecular targeted therapy in glioblastoma. And unexpectedly, we found that IFN-*γ* reduce the expression of CDK4, CDK6, MMP-2, and vimentin, but had no significant impact on the proliferation and migration of glioblastoma cells. The result makes us think deeply. IFN-*γ* inhibits the expression of CDK4, CDK6, MMP-2, and vimentin after significantly upregulating the expression of PD-L1, while the tumor-promoting effect mediated by PD-L1 is also offset.

We speculate that these results may be related to the dual role of IFN-*γ* in tumor immune regulation. A previous study on lung cancer has found that IFN-*γ* inhibits proliferation by activating JAK2/STAT1. The antiproliferative of IFN-*γ* was enhanced by inhibiting PI3K and reduced PD-L1 expression [35]. Although studies have confirmed that IFN-*γ* activates multiple downstream signaling pathways to participate in tumor immune regulation, the mechanism of these signaling pathways in tumor biological behavior is still unclear, and the intersection between these pathways is unknown. In the clinical trial of recombinant IFN-*γ* in cancer treatment, the results showed that the number of patients who benefited was limited, and many patients had serious side effects [36]. Some scholars reported that patients with squamous cell carcinoma of the head and neck, gastric cancer, and metastatic melanoma who were effective against PD-1 had higher expression levels of IFN-*γ*-related genes than ineffective patients [37]. IFN-*γ* signature may be a predictive marker in the treatment of immune checkpoint inhibitors. IFN-*γ* signaling in immune function and tumor immunity is still disputed.

We hypothesized that IFN-*γ* activated antitumor-related signaling pathways while regulating PD-L1 and antagonized the tumor-promoting effect of PD-L1. It is already found that CDK2 and CDK4 play a part in the inhibition of tumor proliferation by IFN-*γ*. In the mouse model, CDK4 and CDK6 knockout allowed the mice to survive [38]. After CDK2 knockout, CDK1 binds to Cyclin E to promote the completion of tumor cell division [39]. Therefore, we hypothesize that there may be compensatory or mutually regulatory effects between cytokines.

## 5. Conclusion

In this research, we identified that IFN-*γ* upregulates the expression of PD-L1 in glioblastoma cells via activating p38/JNK/ERK signaling pathways. PD-L1 enhances the proliferation and migration of glioblastoma cells via regulating CDK4, CDK6, MMP-2, and vimentin molecules. Above all, targeting PD-L1 may be applied to the treatment of glioblastoma. IFN-*γ* counteracts the tumor-promoting effect mediated by PD-L1 in glioblastoma. We speculate that IFN-*γ* may affect glioblastoma through other pathways, and we will continue to further explore its mechanism in the future.

## Figures and Tables

**Figure 1:** PD-L1 expression in human glioblastomas. (a) PD-L1 expression in three human glioblastoma cell lines U251, TG-905, and A172, and two primary cell lines (PT-1 and PT-2) isolated from fresh human surgical glioblastoma tissue samples. (b) IFN-*γ* induced the total protein levels expression of PD-L1 in U251, TG-905, and PT-2, and the effect is the most significant at 24 (h). (c) IFN-*γ* upregulated the surface protein levels expression of PD-L1 in U251, TG-905, A172, PT-1, and PT-2.

**Figure 2:** IFN-*γ* upregulates PD-L1 expression via the p38/JNK/ERK signaling pathways. PD-L1 expression was detected after incubated with SB203580 (a), SP600125 (b), and U0126 (c) in U251, TG-905, and PT-2, prior to IFN-*γ* (50 ng/mL).

**Figure 3:** Eﬃciency of PD-L1 knockdown. (a) PD-L1 mRNA expression in wt group and shRNA-ctl or shRNA-PD-L1 group for U251, TG-905, and PT-2 was detected by qRT-PCR before and after IFN-*γ* stimulation ( ^*∗*^ ^*∗*^ ^*∗*^*P* < 0.001,  ^*∗*^ ^*∗*^ ^*∗*^*P* < 0.001,  ^*∗*^ ^*∗*^*P* < 0.01). (b) PD-L1 protein expression in wt, shRNA-ctl or shRNA-PD-L1 group for U251, TG-905, and PT-2 was detected before and after interferon stimulation.

**Figure 4:** PD-L1 knockdown inhibits glioblastoma cell proliferation. The proliferation capacity of U251 (a) and PT-2 (b) were demonstrated by the CCK8 assay. Compared with shRNA-ctl groups, shRNA-PD-L1 restrained the proliferation of U251 cells (A,  ^*∗*^ ^*∗*^ ^*∗*^*P* < 0.001) and PT-2 cells (B,  ^*∗*^ ^*∗*^ ^*∗*^*P* < 0.001). IFN-*γ* stimulation had no effect on the proliferation of U251 cells (A) and TG-905 cells (B).

**Figure 5:** PD-L1 knockdown inhibits glioblastoma cell migration. A wound-healing assay was implemented on U251 and TG-905 cells at 0, 24, and 48 h after PD-L1 knockdown or IFN-*γ* stimulation. The motility of U251 cells ((a), (b),  ^*∗*^*P* < 0.05) and TG-905 cells ((c), (d),  ^*∗*^*P* < 0.05) in the shRNA-PD-L1 group decreased compared with shRNA-ctl groups. IFN-*γ* stimulation had no effect on the migration of U251 (a) and TG-905 cells (b).

**Figure 6:** Eﬀects of PD-L1 knockdown or IFN-*γ* stimulation on the expression of CDK4, CDK6, MMP-2, vimentin, and GAPDH was tested by western blot in U251 cells.

## Data Availability

The raw data supporting the conclusions of this article will be made available by the authors, without undue reservation.
